RETRACTED

# Dynamic Changes and Influencing Factors for the Quality of Life in Nursing Care after Lung Cancer Resection

**DOI:** 10.1155/2022/1162218

**Published:** 2022-07-31

**Authors:** Shuzhen Hu, Aihong Fang

**Affiliations:** ^1^Department of Cardiothoracic Surgery, Chun'an First People's Hospital, Hangzhou 311700, Zhejiang Province, China; ^2^Department of Surgery, Chun'an Maternity and Child Healthcare Hospital, Hangzhou 311700, Zhejiang Province, China

## Abstract

To investigate the dynamic changes and influencing factors for the quality of life in nursing care in patients with lung cancer after resection. Totally, 136 patients undergoing lung cancer resection in our hospital from January 2019 to January 2022 were prospectively enrolled as subjects. The quality of life was measured before and 1 and 2 weeks and 1, 3, 6, and 12 months after the operation to analyze the dynamic changes in the quality of life in nursing care. Clinical data of patients were collected at the time of discharge. The patients were divided into high-quality and low-quality groups according to the median level of quality of life in nursing care at the final follow-up. The logistic regression equation was applied to analyze the influencing factors for the quality of life in nursing care after lung cancer resection. Of 136 patients receiving lung cancer resection, 32 were lost to follow-up until the final follow-up, so 104 patients were finally included. According to the median level of quality of life in nursing care at the final follow-up, the patients were divided into high-quality and low-quality groups (*n* = 52 per group). The quality of life in nursing care first decreased, then increased, and then stabilized after lung cancer resection. The comparison of clinical data between the two groups exhibited that albumin level was higher in the high-quality group than that in the control group. The age, proportion of living alone, S-AI score, and FoP-Q-SF score were lower in the high-quality group than those in the low-quality group (*P* < 0.05). Univariate logistic regression analysis demonstrated that high albumin (*OR* = 0.884) was a protective factor for the quality of life in nursing care after lung cancer resection (*P* < 0.05). Living alone (*OR* = 1.333), high S-AI score (*OR* = 1.211), high FoP-Q-SF score (*OR* = 1.221), and advanced age (*OR* = 1.209) were the risk factors for the quality of life in nursing care after lung cancer resection (*P* < 0.05). Multivariate logistic regression analysis demonstrated that high albumin (*OR* = 0.861) was a protective factor for the quality of life in nursing care after lung cancer resection (*P* < 0.05). Living alone (*OR* = 1.144), high S-AI score (*OR* = 1.170), high FoP-Q-SF score (*OR* = 1.161), and advanced age (*OR* = 1.181) were the risk factors for the quality of life after lung cancer resection (*P* < 0.05). The quality of life in nursing care first decreased, then increased, and then stabilized after lung cancer resection. Albumin, age, living alone, and S-AI and FoP-Q-SF scores were the influencing factors for the quality of life in nursing care after lung cancer resection. In the nursing care process after lung cancer resection, we should focus on elderly patients living alone who are affected by anxiety and fear of recurrence to improve the quality of life of these patients.

RETRACTED

## 1. Introduction

Lung cancer is the most rapidly increasing malignancy with an incidence rate in our country of over 30 years. The results of our second cause of death sampling survey show that lung cancer mortality has ranked the third leading cause of death from cancer in the 1990s, second only to gastric and esophageal cancer. The third cause of death retrospective survey in the 21st century revealed that lung cancer has become the leading cause of death from cancer. Data released by the National Cancer Center in 2016 showed that in 2015, there were 733 000 new cases of pulmonary blast in China (5093 000 males and 2240 000 females), ranking first among malignant tumors (20.27% males and 12.59% females), accounting for 17.09% of new cases of malignant tumors (20.27% males and 12.59% females) · during the same period, there were 6102 000 lung cancer deaths in China (4324 000 males and 1778 000 females), accounting for 21.68% of deaths due to malignant tumors (23.89% males and 17.70% females). Geographically, the mortality rate of lung cancer in urban China is higher than that in rural areas. The mortality rate of lung cancer is significantly higher in urban and rural areas in East and central China than in the West. The mortality rate is rapidly increasing in people with an onset age > 40 years.

Lung cancer is an extensive type of malignant tumor worldwide. Despite remarkable progress in multidisciplinary treatment, surgery is still the preferred treatment for patients with resectable lung cancer when the patients can physically tolerate lung cancer resection. It can effectively remove diseased tissue and improve outcomes and postoperative quality of life [1]. Nevertheless, a study has shown the differences in the early and long-term quality of life changes in some patients after lung cancer resection [2]. The quality of life is an index to comprehensively assess the patient's condition after lung cancer resection and can fully reflect the surgical effect and health status. Good quality of life predicts good outcomes for the patient. The quality of life has been regarded as a crucial outcome indicator after lung cancer resection, especially in nursing-related studies [3, 4]. Therefore, effectively assessing the quality of life and grasping the dynamic change rule and influencing factors of the quality of life will help medical staff to master the patient's condition and to assess the outcomes after lung cancer resection and will also help nursing staff to provide high-quality nursing services.

RETRACTED

In recent years, research on influencing factors of quality of life of lung cancer mainly focuses on demographic and sociological characteristics (age, gender, marital status, ethnicity, residence, work situation, and economic status), disease characteristics (staging, classification, surgical method, scope of surgery, and adjuvant treatment), depression, health status (smoking status, body mass index, and complications). In contrast, our domestic studies mainly covered the following topics: gender, age, educational background, surgical method, personal income, time of diagnosis, marital status, comorbidities, and CO diffusion capacity. In the study by Jin et al. [5], age and sex were considered the major factors leading to differences in the quality of life data after lung cancer resection. However, a cross-sectional study by Codima et al. [6] confirmed the differences in the quality of life after the same type of lung cancer resection and indicated that there may be other potential influencing factors affecting the quality of life after lung cancer resection. To determine the dynamic changes and the influencing factors for the quality of life of patients undergoing lung cancer resection, this study discussed the dynamic changes and influencing factors for the quality of life in nursing care after lung cancer resection.

## 2. Materials and Methods

### 2.1. Research Subjects

After approval by the hospital ethics committee, 136 patients undergoing lung cancer resection in our hospital from January 2019 to January 2022 were prospectively recruited as subjects. Inclusion criteria are as follows: (1) first onset of primary nonsmall cell lung cancer; (2) receiving lung cancer resection, clinical stages I-II; (3) postoperative adjuvant chemotherapy; (4) patients and their families signed informed consent. Exclusion criteria: (1) combination with other tissue or organ tumors, cognitive dysfunction, and history of cerebrovascular disease; (2) the patients cannot take care of themselves because of the combination with muscle, joint, and bone diseases; (3) poor compliance. Exclusion criteria are as follows: (1) Request to withdraw from these study midway; (2) patients who died or were lost to follow-up; (3) patients with other symptoms affecting this study.

RETRACTED

### 2.2. Research Methods

#### 2.2.1. Research Ideas

Totally 136 patients receiving lung cancer resection in our hospital from January 2019 to January 2020 were recruited in this study. The quality of life was measured before, 1 and 2 weeks, 1, 3, 6, and 12 months after the operation. The dynamic changes in the quality of life were analyzed and clinical data of patients at discharge were collected. The patients were divided into high-quality and low-quality groups according to the median level of quality of life in nursing care at the final follow-up. The Logistic regression equation was employed to analyze the influencing factors for the quality of life in nursing care after lung cancer resection.

#### 2.2.2. Data Collection

The general data of all patients were obtained when they were discharged from the hospital, containing age, sex, BMI, clinical-stage, complication, living alone, metastasis, surgical methods, adjunctive therapy, laboratory test indicators, and psychological status. Simultaneously, the quality of life of patients was detected before, 1 and 2 weeks, 1, 3, 6, and 12 months after the operation.

#### 2.2.3. Laboratory Examination Indicators

Totally 5 mL of fasting peripheral venous blood harvested from patients was maintained at room temperature for 30 minutes and centrifuged at 3000 r/min and 4°C for 15 minutes. The supernatant was placed in a −80°C refrigerator for testing. A biochemical analyzer (Beckman Coulter, AU5800, US) was utilized to examine serum creatinine, alanine aminotransferase, albumin, and serum CEA. Arterial blood was harvested from patients to measure PaO_2_ and PaCO_2_ using a Stat Pm6le pHOx blood gas analyzer.

#### 2.2.4. Quality of Life Measurement

The quality of life of patients was measured by using the Chinese version of the European Organization for Research and Treatment of Cancer (EORTC) QLQ-C30 form in the evaluation of the quality of life for patients with cancer [7] before, 1 and 2 weeks, 1, 3, 6, and 12 months after surgery. This form has 30 items, containing 5 functioning scales (physical/emotional/cognitive/social/role), 9 symptom scales (fatigue/nausea and vomiting/pain/dyspnea/insomnia/appetite loss/constipation/diarrhea/financial difficulties) and Global Health Status Scale scores, totally 15 domains. In this study, only the Global Health Status Scale score was counted, with a score ranging from 0 to 100. The higher the score, the better the quality of life is.

#### 2.2.5. Psychological State

State-trait anxiety inventory (S-AI) [8] was utilized to assess the patient's anxiety state when the patient was discharged from the hospital. This scale has 20 items, using the 4-point Likert scale (1 point to 4 points), with a total score of 80. The higher the score, the more obvious the patient's anxiety is. The Chinese version of the Fear of Progression Questionnaire-Short Form (FoP-Q-SF) [9]was employed to measure fear of recurrence. This scale has 12 items, using the 5-point Likert scale, with a total score of 12 to 60. The higher the score, the higher the degree of fear of recurrence is.

RETRACTED

### 2.3. Statistical Methods

All data were analyzed using SPSS 22.0 statistical software. The measurement data that met the normal distribution were represented by the mean ± standard deviation. The comparison between groups was performed by an independent-sample *t*-test. The measurement data that did not meet the normal distribution were expressed by the median (quartile) method and the Mann-Whitney *U* test was applied. The count data were expressed by *n*(%) and the *x*^2^ test was used. Multivariate analysis was performed using a Logistic regression equation. A value of *P* < 0.05 was considered statistically significant.

## 3. Results

### 3.1. Follow-Up Results

Of 136 patients undergoing lung cancer resection, 32 patients were lost to follow-up until the final follow-up, so 104 patients were finally included. According to the median level of quality of life in nursing care at the final follow-up (67 points), the patients were assigned to high-quality and low-quality groups (*n* = 52 per group).

### 3.2. Dynamic Analysis of the Quality of Life of Patients after Lung Cancer Resection

The quality of life of patients with lung cancer first decreased, then increased, and then stabilized after lung cancer resection, as shown in Table 1 and Figure 1.

### 3.3. Comparison of Clinical Data of the Two Groups

As shown in Table 2, clinical data comparing the two groups were available, except that the albumin level was higher in the high-quality group than in the low-quality group (*P* < 0.001). Age, proportion living alone, S-AI score, and FoP-Q-SF score were lower in the high-quality group than in the low-quality group (*P* < 0.05).

### 3.4. Univariate Logistic Analysis of Factors Affecting the Quality of Life in Nursing Care after Lung Cancer Resection

Univariate Logistic regression analysis displayed that high albumin (*OR* = 0.884) was a protective factor for the quality of life in nursing care after lung cancer resection (*P* < 0.05). Living alone (*OR* = 1.333), high S-AI score (*OR* = 1.211), high FoP-Q-SF score (*OR* = 1.221), and advanced age (*OR* = 1.209) were risk factors for the quality of life in nursing care after lung cancer resection (*P* < 0.05), as shown in Table 3.

RETRACTED

### 3.5. Multivariate Logistic Analysis of Factors Affecting the Quality of Life in Nursing Care after Lung Cancer Resection

Multivariate Logistic regression analysis demonstrated that high albumin (*OR* = 0.861) was a protective factor for the quality of life in nursing care after lung cancer resection (*P* < 0.05). Living alone (*OR* = 1.144), high S-AI score (*OR* = 1.170), high FoP-Q-SF score (*OR* = 1.161), and advanced age (*OR* = 1.181) were risk factors for the quality of life in nursing care after lung cancer resection (*P* < 0.05), as shown in Table 4.

## 4. Discussion

Lung cancer is a chief cause of cancer-related death worldwide. Surgery, a major way to treat lung cancer, can effectively improve clinical symptoms and prolong the life span [10]. In addition to the improvement of clinical symptoms, which can be used as an evaluation index for the efficacy of surgical treatment, the quality of life is also an outcome index for lung cancer patients after lung cancer resection [11]. Steffens et al. [12] stated that the quality of life after lung cancer resection can comprehensively reflect the changes in health status and severity and is a strong predictor of outcomes. Taken together, it is of great significance for patients and their nursing staff to improve the quality of nursing care by grasping the quality of life of patients after lung cancer resection. Nevertheless, the results from a previous study concerning the alteration in the quality of life in the first year after lung cancer resection are conflicting [13]. Moreover, the research addressing the influencing factors for the quality of life after lung cancer resection mainly focuses on age, complication, and surgical methods [13]. However, a study has shown that its predictive performance is not good and indicated that there may be other factors affecting the quality of life after lung cancer resection [14]. To find out the influencing factors for the quality of life 1 year after lung cancer resection, this study enrolled 136 patients undergoing lung cancer resection to investigate the influencing factors for the quality of life.

The results from the present study confirmed that the quality of life in nursing care first decreased, then increased, and then stabilized after lung cancer resection, indicating that the quality of life is a dynamic process. It is concluded that the decrease in quality of life in the early postoperative period, especially within one month after surgery, was associated with surgical trauma, pain, immobilization, and early postoperative fatigue. In a study by Ichimura et al. [15] on survivors after lung cancer surgery, it was found that postoperative quality of life decreased in approximately 73% of patients due to surgical trauma and pain and approximately 51% of patients could not complete daily life independently due to postoperative immobilization and fatigue. Some scholars have proposed that a high health-related quality of life can be achieved by adjusting the analgesic regimen, adding physical training after lung cancer resection, reducing pain, and diminishing the incidence of postoperative fatigue [16]. The results from the current study verified that the quality of life gradually increased and then stabilized at 3, 6, and 12 months after surgery. It might be that with the prolongation of time, the pain and immobilization caused by surgical trauma were relieved; with the implementation of subsequent adjuvant therapy and functional exercise, lung function, mobility, and functional level gradually recovered in patients receiving lung cancer resection. Thus, the quality of life gradually improves. It was also found in a meta-analysis that the quality of life of 75–93% of patients gradually recovered 3–9 months after surgery [17]. Although the psychological trauma suffered by cancer patients can be mitigated over time, most patients still have adverse psychological conditions such as fear of recurrence, which may limit the further improvement of quality of life to a certain extent. Lim et al. [18] also pointed out that more than half of the patients after lung cancer resection have suffered from adverse psychological states such as fear of recurrence, which can limit further recovery of the quality of life to a certain degree.

RETRACTED

Univariate and multivariate Logistic regression analyses in this study demonstrated that high albumin was a protective factor for the quality of life in nursing care after lung cancer resection. These analyses have verified that the albumin level reflects the nutritional status and a low albumin level indicates a poor nutritional status. However, a large number of nutrients need to be consumed to repair surgical trauma and body functions during the recovery after lung cancer resection. The poor nutritional status can result in muscle mass loss and energy deposition consumption, so it is difficult for patients to perform daily activities, which reduces personal strength and autonomy and in turn, decreases the quality of life. Klimczak et al. [19] studied the relationship between nutritional status and quality of life in patients with nonsmall cell lung cancer and found that malnourished nonsmall cell lung cancer patients presented a low quality of life. Nutritional support to patients with advanced nonsmall-cell lung cancer during chemotherapy can effectively improve their nutritional status, reduce the incidence of toxic and side effects, and improve the tolerance of patients, improve their quality of life. Regarding negative emotions, the mental state of elderly patients with malignant tumors is worse than that of young and middle-aged patients, especially elderly patients with malignant tumors living alone [20]. This study draws similar conclusions that living alone, high S-AI score, high FoP-Q-SF score, and advanced age are risk factors for the quality of life in nursing care after lung cancer resection. During the long-term treatment after discharge from the hospital, living alone can increase loneliness and anxiety. The physiological decline in body functions increases patients' frustration. During this negative emotion, the anxiety, fear, and worry about the disease have no one to tell and cannot be enlightened, which promotes further development of negative emotions. Simultaneously, the feeling, understanding of social support, and the ability to understand social support are reduced in elderly patients receiving lung cancer resection who live alone, thus forming a vicious circle, which may finally affect the treatment compliance and willingness and worsen the quality of life. A prospective study by Sommer et al. [21] also concluded that with prolonged time, the correlation of anxiety and fear of recurrence with living alone and age gradually increased in patients receiving lung cancer resection and that the age, living alone, anxiety, and fear of disease recurrence are independent influencing factors for the quality of life in nursing care after lung cancer resection, confirming the effects of age, living alone, anxiety, and fear of recurrence on the quality of life after lung cancer resection.

RETRACTED

## 5. Conclusion

In conclusion, the quality of life of nursing care after resection for lung cancer first decreased, then increased, and then stabilized. High albumin is a protective factor for the quality of life after lung cancer resection. Advanced age, living alone, and high S-AI and FoP-Q-SF scores were risk factors for the quality of care after lung cancer resection. In the process of care, we should focus on elderly patients living alone, who have anxiety and fear of recurrence, to improve the quality of life of these patients. The limitation of this study is that it was a single-center small sample study. Meanwhile, quality of life changes dynamically during long-term follow-up after lung cancer resection, and the influencing factors may be different at each time point. This study only investigated the correlation between clinical data at discharge and quality of life at final follow-up, so our results may be biased. Soon, multicenter large sample studies should be performed. Clinical data and quality of life should be dynamically analyzed to further explore the influencing factors on quality of life after lung cancer resection.

## Figures and Tables

**Figure 1:** Dynamic analysis of the quality of life of patients after lung cancer resection.

**Table 1:** Dynamic analysis of the quality of life of patients receiving lung cancer resection ($\bar{x}$ ±*s*, points).

Index	Before surgery	1 week after surgery	2 weeks after surgery	1 month after surgery	3 months after surgery	6 months after surgery	12 months after surgery
Quality of life	70.14 ± 15.87	42.62 ± 9.65	35.32 ± 11.40	48.62 ± 9.84	67.32 ± 12.58	73.84 ± 10.58	74.86 ± 10.19

**Table 2:** Comparison of clinical data of the two groups (($\bar{x}$ ± *s*)/*n*(%)).

Index	Low-quality group (*n* = 52)	High-quality group (*n* = 52)	*Z/t/χ * ^2^	*P*
Age (year)	68.71 ± 5.66	59.57 ± 6.67	5.892	<0.001
Sex (male/female)	34/18	26/26	2.521	0.112
BMI (kg/m^2^)	23.12 ± 2.14	24.01 ± 2.49	−1.955	0.053

Complication (*n*(%))				
Hypertension	11 (21.15)	9 (17.31)	0.248	0.619
Diabetes	8 (15.38)	6 (11.54)	0.330	0.566
Hyperlipidemia	6 (11.54)	2 (3.85)	2.167	0.141

Clinical stage (*n*(%))			1.493	0.222
I	16 (30.77)	22 (42.31)		
II	36 (69.23)	30 (57.69)		
Living alone (*n*(%))	16 (30.77)	4 (7.69)	8.914	0.003
Metastasis (*n*(%))	19 (36.54)	(40.38)	0.163	0.687

Surgical methods (*n*(%))			0.768	0.443
Lobectomy	15 (28.85)	11 (21.15)	0.242	0.623
Segmental resection	16 (30.77)	17 (32.69)	1.083	0.298
Wedge resection	21 (40.38)	24 (46.15)	3.581	0.058

Adjuvant therapy (*n*(%))			0.977	0.329
Radiotherapy	11 (21.15)	14 (26.92)		
Chemotherapy	34 (65.38)	35 (67.31)		
Others	7 (13.46)	3 (5.77)		
S-AI (point)	54.10 ± 7.96	42.70 ± 7.66	7.442	<0.001
FoP-Q-SF (point)	37.70 ± 6.10	29.86 ± 7.14	6.019	<0.001
Serum CEA (ng/mL)	44.87 ± 8.43	46.26 ± 9.75	0.778	0.439
Serum creatinine (*μ*mol/L)	59.89 ± 11.51	61.47 ± 10.32	0.737	0.463
Alanine aminotransferase (U/L)	30.11 ± 5.89	31.76 ± 5.25	1.508	0.135
Albumin (g/L)	57.11 ± 10.04	71.79 ± 12.24	6.688	<0.001
PaO_2_ (mmHg)	92.57 ± 10.45	96.31 ± 11.96	1.698	0.093
PaCO_2_ (mmHg)	40.96 ± 3.85	39.93 ± 3.54	1.420	0.159

**Table 3:** Univariate logistic analysis on factors affecting the quality of life in nursing care after lung cancer resection.

Related indicators	*β*	*S.E*	*Wald*	*P*	*OR*	95% C.I.	
						Lower limit	Upper limit
Living alone	1.674	0.601	7.760	0.005	1.333	1.042	1.378
S-AI score	0.191	0.039	24.599	0.000	1.211	1.123	1.306
FoP-Q-SF score	0.200	0.045	19.854	0.000	1.221	1.119	1.334
Albumin	−0.124	0.026	23.007	0.000	0.884	0.840	0.929
Age	0.19	0.042	20.839	0.000	1.209	1.115	1.312

RETRACTED

**Table 4:** Multivariate logistic analysis on factors affecting the quality of life in nursing care after lung cancer resection.

Related indicators	*β*	*S.E*	*Wald*	*P*	*OR*	95% C.I.	
						Lower limit	Upper limit
Living alone	2.317	1.223	3.587	0.048	1.144	1.022	1.548
S-AI score	0.157	0.054	8.387	0.004	1.170	1.052	1.301
FoP-Q-SF score	0.15	0.069	4.713	0.030	1.161	1.015	1.329
Albumin	−0.15	0.042	12.679	0.000	0.861	0.792	0.935
Age	0.167	0.063	7.098	0.008	1.181	1.045	1.336
Constant	−14.492	5.221	7.705	0.006			

## Data Availability

The simulation experiment data used to support the findings of this study are available from the corresponding author upon request.
